# Paeoniflorin Protects H9c2 Cardiomyocytes against Hypoxia/Reoxygenation Induced Injury via Regulating the AMPK/Nrf2 Signaling Pathway

This article has been retracted.

**DOI:** 10.1155/2022/7667770

**Published:** 2022-10-13

**Authors:** Wen Yu, Huang Sun, Yang Tan, Wei Zhang

**Affiliations:** ^1^Department of Emergency, The First Affiliated Hospital of Kunming Medical University, 295 Xichang Road, Kunming, Yunnan, China; ^2^Department of Cardiology, The First Affiliated Hospital of Kunming Medical University, 295 Xichang Road, Kunming, Yunnan, China

## Abstract

Myocardial ischemia/reperfusion (MIR) injury contributes to the exacerbation of heart disease by causing cardiac arrhythmias, myocardial infarction, and even sudden death. Studies have found that paeoniflorin (PF) has a protective effect on coronary artery disease (CAD). However, the mechanism of PF in MIR has not been fully investigated. The purpose of this study was to investigate the functional role of PF in H9c2 cells subjected to hypoxia/reoxygenation (H/R). Here, PF treatment enhanced cell viability in H/R-stimulated H9c2 cells. In H9c2 cells, PF treatment reduced the formation of reactive oxygen species (ROS) induced by H/R. In H/R-stimulated H9c2 cells, PF also increased the activity of antioxidant enzymes such as superoxide dismutase and glutathione peroxidase. Furthermore, PF protected H9c2 cells against H/R-induced apoptosis, as demonstrated by increased Bcl-2 expression, decreased Bax expression, and decreased caspase-3 activity. Furthermore, PF increased the levels of p-AMPK and nuclear Nrf2 expression in response to H/R stimulation. AMPK inhibition, on the other hand, abolished the PF-mediated increase in Nrf2 signaling and the cardiac-protective effect in H9c2 cells exposed to H/R. These data suggest that PF protected H9c2 cells against H/R-induced oxidative stress and apoptosis through modulating the AMPK/Nrf2 signaling pathway. Our findings support the therapeutic potential of PF in myocardial I/R damage.

## 1. Introduction

Myocardial infarction is a common fatal and disabling disease [1]. Myocardial ischemia is caused by coronary artery obstruction or stenosis, resulting in insufficient myocardial blood supply, the imbalance between cardiac oxygen supply and oxygen demand, resulting in loss of myocardial cells and the formation of cardiac scar, ultimately leading to heart failure [2]. However, myocardial ischemia-reperfusion injury (MIR) often occurs after treatment of this disease, which leads to the death of a large number of myocardial cells and aggravation of myocardial injury [3]. At present, platelet regulation drugs, *β*–blockers, and calcium channel antagonists are used to treat this disease clinically [4–6]. Although modern medicine has made great progress in the treatment of myocardial ischemia, there are no effective drugs. Therefore, prevention and treatment of myocardial ischemia-reperfusion injury is an effective method to treat myocardial infarction. The pathophysiological mechanism of myocardial ischemia-reperfusion injury is complex. Studies have shown that myocardial ischemia can promote inflammation and oxidative stress translation and can lead to myocardial apoptosis through reperfusion, in which inflammatory factors can activate and chemotaxis leukocytes, which are also the products of activation of the leukocytes, which can aggravate myocardial injury [1, 7–9]. Superoxide dismutase (SOD) is essential to prevent oxidative stress, and it can effectively resist the damage of oxygen free radicals to the body through its antioxidant and antifree radical functions [10]. The surface level of malondialdehyde (MDA) in the body can reflect the level of oxygen free radicals in the body, and then, reflect the damage degree of oxidative stress in the body [11]. Therefore, oxidative stress plays an important role in the occurrence and development of myocardial ischemia-reperfusion injury.

Paeoniflorin (PF) is a bioactive glycoside isolated from the root of Paeonia Alba. Paeoniflorin has been reported to have beneficial effects on the cardiovascular system (hypertension, atherosclerosis, and bleeding) and the nervous system (headaches, vertigo, dementia, and pain) [12]. Paeoniflorin by lowering lipid peroxidation products MDA and ROS generation level, reducing oxidative stress, and increase the glutathione (GSH) content, thus, reducing oxidative stress and inflammatory pathways, effectively avoiding the loss of neurons and microglia activation and cerebral white matter lesions, which caused by hypoxia-ischemia brain damage to play effective protection [12–14]. Previous studies showed that the mechanism of PF's ability to exert antioxidative stress injury may be related to improving the activity of SOD and other antioxidant enzymes in vivo, thus, alleviating the damage of oxygen free radicals to the body [15]. The effects of PF on I/R-mediated oxidative stress and apoptosis in cardiomyocytes, on the other hand, are unknown.

In this study, the hypoxia/reoxygenation injury model of myocardial cells was used to simulate the ischemic injury of ischemic heart disease in the process of hypoxia and the reperfusion injury in the process of reoxygenation after hypoxia. The levels of creatine kinase muscle/brain (CK-MB), lactate dehydrogenase (LDH), and MDA in cell culture medium at different time points during hypoxia/reoxygenation were measured to evaluate the degree of damage to myocardial cells, and then to evaluate the protective effect and mechanism of PF on hypoxia/reoxygenation injury of myocardial cells.

## 2. Materials and Methods

### 2.1. Cell Culture

The rat cardiomyocyte-derived H9c2 cell line was purchased from the cell bank of the Chinese Academy of Sciences. The H9c2 cells were gown in Dulbecco's modified Eagle's medium, added with 10% FBS at 37 in a 5% CO_2_ atmosphere.

### 2.2. Establishment of Hypoxia/Reoxygenation (H/R) Model [16]

H9c2 cells were cultivated in a hypoxic environment with 1% O_2_, 94% N_2_, and 5% CO_2_ in modular gas chambers for 24 h, and then, reoxygenated for 2 h at 37 C in a 21% O_2_, 5% CO_2_, and 74% N_2_ incubator. Before H/R stimulation, cells were pretreated with or without PF for 2 h.

### 2.3. Cell Viability Assay

The 3-(4, 5-dimethylthiazol)-2, 5-diphenyltetrazolium bromide (MTT) assay kit was used to analysis cell viability. H9c2 cells were seeded in 96-well plates and grown for 24 h prior to H/R. H9c2 cells were cultured for 1 h with 10 ul MTT solution following various treatments. Then, the H9c2 cells were added with 200 ml of DMSO to dissolve the formazan crystals. A microplate reader (Varioskan Flash, Thermo, Finland) was measured to measure absorbance at 490 nm, and the absorbance values of control cells were adjusted to 100%.

### 2.4. Cell Cytotoxicity Assay

The culture supernatants were collected after 24 h of incubation with various concentrations of PF (0, 5, 10, 20, and 40 mM) to determine lactate dehydrogenase (LDH) leakage. The LDH detection kit was used to analyze the LDH content.

### 2.5. Measurement of Cellular ROS Production

Flow cytometry was used to examine the generation of intracellular ROS using dichlorofluorescin diacetate as the fluorescent probe. In brief, H9c2 cells were washed with PBS before being treated with 10 mM DCFH-DA at 37 for 30 min in the dark. The flow cytometer was then used to investigate H9c2 cells using a 488 nm excitation filter and a 525 nm emission filter.

### 2.6. Determination of SOD, MDA, and GSH

H9c2 whole cell lysates were collected according to the manufacturer's instructions using RIPA lysis buffer. The activities of SOD, MDA, and GSH were investigated using the corresponding kits. The MDA level was determined using the thiobarbituric acid method and MDA detection kit (A003-1-2; Jiancheng Bioengineering Institute). SOD and GSH activity were detected using the hydroxylamine method, and total SOD detection kit, and GSH detection kit (Jiancheng Bioengineering Institute).

### 2.7. Western Blot Analysis

Cells were washed with precooled PBS and added to the protein lysate. The supernatant was removed and obtained after centrifugation. The protein content was determined by the BCA method. Mix with protein loading buffer in proportion, heat at 100 to denaturate protein, and store at low temperature for later use. The proteins in the polyvinylidene fluoride (PVDF) gel were transferred to a polyvinylidene fluoride (PVDF) membrane by sodium dodecyl sulfate and polyacrylamide gel electrophoresis, and were sealed at 5% BSA at room temperature for 2 h. The B cell lymphoma-2 (Bcl-2), Bax, Caspase3, P-AMPK, AMPK, Nrf2, GAPDH, and lamin B2 primary antibody (Abcam) were added to a resistant shaker overnight. The PVDF membrane was washed by TBST for 3 times, 5 min each time, and placed into the rat secondary antibody (1 : 5000) for incubation for l ∼ 2 h. The PVDF membrane was removed and washed by TBST for 3 times, 5 min each. The ECL kit was used for development, the chemiluminescence gel system analyzer was used for display, and photos were taken using VisionWorks 6.3.3. The gray values of protein bands were analyzed by image acquisition and analysis software with GAPDH as an internal reference. The experiment was repeated three times. The images were scanned for preservation and analyzed with ImageJ software, with the gray-scale value digitized on each special band.

### 2.8. Caspase-3 Activity

Caspase-3 activity of H9c2 cells was analyzed by using a Caspase-3 Colorimetric Assay Kit. In brief, H9c2 cell lysates were treated at 37 with caspase 3 substrates, Ac-DEVD-pNA and the released p-NA was quantified using a spectrophotometer at 405 nm.

### 2.9. Statistical Analysis

Graphpad software was used to analyze the results of three separate tests, which were reported as mean + SD. One-way ANOVA was used to assess group comparisons, followed by the least significant difference test. *P* < 0.05 was considered to be statistically significant. ^*∗*^*P* < 0.05 denotes a significant change as compared to control H9c2 cells. #*P* < 0.05 denotes a significant change as compared to H9c2 cells treated with H/R. ^$^*P* < 0.05 denotes a significant difference when compared to the H/R + PF groups.

## 3. Results

### 3.1. PF Improves the Cell Viability and Injury in H/R Stimulated H9c2 Cells

To explore the effect of PF on H/R stimulated H9c2 cells, the cells were incubated with a series of concentration of PF (0, 50, 100, and 200 *μ*M) for 24 h. The MTT assay demonstrated that H/R inhibited H9c2 cell viability. The different concentrations of PF (50, 100, and 200 *μ*M) treatments markedly enhanced the cell viability in H/R induced H9c2 cells (Figure 1(a)). LDK leakage assay showed that H/R increased the LDK leakage and the different concentration of PF (50, 100, and 200 *μ*M) treatments markedly decreased the LDK leakage in H/R induced H9c2 cells (Figure 1(b)). Besides, the H/R induced the production of CK-MB and the different concentration of PF (50, 100, and 200 *μ*M) treatments reduced the CK-MB level in H/R induced H9c2 cells (Figure 1(c)). Therefore, PF effectively protected the cell viability and injured H/R stimulated H9c2 cells.

### 3.2. PF Represses Oxidative Stress in H9c2 Cells Exposed to H/R Treatment

As shown in Figure 2(a), the ROS level was higher in the H/R group than control, while PF markedly decreased the production of ROS in H/R stimulated H9c2 cells. Moreover, the activity of SOD and GSH were reduced in H/R group compared with control, PF markedly enhanced the SOD and GAH activities (Figures 2(b) and 2(c)); H/R-induced increase in the MDA activities, which was blocked by pretreatment with PF (Figure 2(d)). Thus, PF reduces oxidative stress in H9c2 cells exposed to H/R.

### 3.3. PF Inhibits Apoptosis in H9c2 Cells Exposed to H/R Treatment

Subsequently, cell apoptosis was assessed by detecting the expression levels of Bax and Bcl-2. As shown in Figures 3(a)–3(c), H/R treatment significantly increased the Bax protein expression and reduced the Bcl-2 protein expression in H9c2 cells, while PF prevented the change of Bax and Bcl-2 protein caused by H/R. In addition, the caspase-3 activity was significantly enhanced in H/R stimulated H9c2 cells; PF markedly inhibited the caspase-3 activity in H/R stimulated H9c2 cells (Figure 3(d)). Thus, PF reduced cell apoptosis in H9c2 cells exposed to H/R treatment.

### 3.4. PF Induced the Activation of AMPK/Nrf2 Signaling Pathway

The AMPK/Nrf2 signaling pathway has been discovered as a ROS-activated antioxidant signaling mechanism. We then looked at how PF affected AMPK/Nrf2 activation in H/R-exposed H9c2 cells. As shown in Figures 4(a)–4(c), the levels of p-AMPK and nuclear Nrf2 were inhibited in H/R-exposed H9c2 cells, PF increased the levels of p-AMPK, and nuclear Nrf2 in H/R-exposed H9c2 cells.

### 3.5. Treatment with Compound C Reserved the Effects of PF on Cell Viability, Oxidative Stress, and Apoptosis in H/R Stimulated H9c2 Cell

Compound C, an AMPK inhibitor, was employed to impede AMPK signaling in order to validate the involvement of AMPK/Nrf2. Compound C treatment resulted in the predicted reduction in nuclear Nrf2 expression in H9c2 cells (Figures 5(a)–5(c)). Furthermore, AMPK inhibition effectively reversed the regulatory effects of PF on cell survival (Figure 5(d)), ROS levels (Figure 5(e)), and caspase-3 activity (Figure 5(f)). These findings revealed that AMPK mediated the role of PF on Nrf2 signaling in H9c2 cells.

## 4. Discussion

At present, the basic treatment principle for ischemic heart disease is to restore reperfusion. The recovery of reperfusion not only improves the ischemic state, but also causes myocardial injury again–reperfusion injury. Myocardial cell hypoxia/reoxygenation model well simulated myocardial cell reperfusion injury [17]. It is generally believed that during hypoxia/reoxygenation, cardiomyocytes produce various oxygen free radicals, which react with the peroxidation of cell membrane and biological macromolecules and destroy the normal structure of the cell membrane [18]. Myocardial enzymes such as CK and LDH leak out of the cell with the destruction of the cell membrane, and the peroxide MDA of membrane lipid molecules is produced in large quantities, resulting in the lack of reoxygenation injury of cardiomyocytes [19]. Therefore, myocardial cell injury is the culprit of myocardial ischemia and ischemia-reperfusion injury, and the key to the treatment of such diseases is to combat myocardial cell injury. In this study, the H/R induced the production of CK-MB, and the different concentrations of PF (50, 100, AND 200 *μ*M) treatments reduced the CK-MB level in H/R induced H9c2 cells. Therefore, PF effectively protected the cell viability and injured H/R stimulated H9c2 cells.

The caspase family is an important molecule that mediates cell apoptosis. Caspase-3 and Caspase-9 are involved in signal transduction of the death receptor apoptosis pathway and mitochondrial apoptosis pathway, respectively [20]. Finally, caspase-3 is activated and apoptosis is performed through cascade activation of multiple downstream caspase molecules [21, 22]. Paeoniflorin is the active ingredient of Paeonia lactiflora, which can protect cells from inflammation and oxidation [23]. In order to define the paeoniflorin effects on myocardial ischemia injury in the process of apoptosis, we measured caspase-3 activity and apoptosis gene expression quantity on the basis of the comparison. The results showed that paeoniflorin H9c2 cells in ischemia reperfusion, so paeoniflorin can inhibit myocardial ischemia injury in the process of cell apoptosis, and alleviate myocardial damage.

The nuclear factor E2-related factor 2 (Nrf2) is a key transcription factor widely existing in animals to defend against oxidative stress and can combine with antioxidant response elements (ARE) to activate downstream antioxidant genes, such as HO-1 and NQO1, so as to resist various protoplasts-induced intracellular oxygenation excitation states [24, 25]. Adenosine monophosphate-activated protein kinase (AMPK), a silk/threonate albuminase composed of three peptide chains, is an important regulator of human energy metabolism and is closely related to promoting catabolism, inhibiting anabolism, improving endothelial function, alleviating inflammatory response, and inhibiting oxygen-reduction reaction [26, 27]. It has been shown in previous studies that AMPK can activate Nrf2 through phosphorylation and generate downstream antioxidant genes such as HO-1 and NQO1 to play an antioxidative stress role [28]. Here, we found that PF induced the activation of the AMPK/Nrf2 signaling pathway in H/R stimulated H9c2 cells.

A previous study reported that Galanthamine improves myocardial I/R induced cardiac dysfunction by activating the AMPK/Nrf2 pathway in rats [29]. Galanthamine improves myocardial I/R-induced cardiac dysfunction by activating AMPK/Nrf2 pathway in rats [28]. Galanthamine improves myocardial I/R-induced cardiac dysfunction by activating the AMPK/Nrf2 pathway in rats [30]. Here, we found that PF induced the activation of the AMPK/Nrf2 signaling pathway in H/R stimulated H9c2 cells. Compound C, an AMPK inhibitor, was employed to impede AMPK signaling in order to validate the involvement of AMPK/Nrf2. AMPK inhibition dramatically reversed the regulatory effects of PF on cell survival, ROS levels, and caspase-3 activity. These findings revealed that AMPK mediated the control of PF on Nrf2 signaling in H9c2 cells.

## 5. Conclusions

In conclusion, our findings show that PF protects H/R stimulated H9c2 cells by inhibiting oxidative stress and apoptosis. The AMPK/Nef2 signaling pathway was activated to control the protective effects of PF. As a result, PF might be a potential therapeutic medication for the treatment of myocardial I/R damage.

## Figures and Tables

**Figure 1:** Effect of PF on cell viability, LDK and CK-MB level in H/R induced H9c2 cells. H9c2 cells were added with PF (50, 100, 200 *μ*M) for 2 h and then subjected to H/R stimulation. (a) MTT assay was used to analyze the cell viability. (b) LDK leakage assay was used to assess the cytotoxic effect of PF in H9c2 cells. (c) ELISA was performed to assess the CK-MB levels in H9c2 cells. *N* = 3, ^*∗*^*P* < 0.05 vs. control. #*P* < 0.05 vs. H/R.

**Figure 2:** Effect of PF on oxidative stress in H9c2 cells. (a) Flow cytometry was used to assess ROS generation in H9c2 cells. (b–d) SOD, GSH, and MDA activities in H9c2 cells were measured by ELISA. *N* = 3, ^*∗*^*P* < 0.05 vs. control. #*P* < 0.05 vs. H/R.

**Figure 3:** PF's effect on apoptosis in H9c2 cells. (a) Western blot analysis was used to determine the levels of expression of apoptosis-related proteins such as bax and bcl-2. Quantification of bax and bcl-2 (b and c). The caspase-3 activity with the substrate peptide Ac-DEVD-pNA was measured using a colorimetric technique (d).

**Figure 4:** The effect of PF on the AMPK/Nrf2 signaling pathway in H9c2 cells activated with H/R. (a) Western blot was used to determine the levels of AMPK, p-AMPK, and nuclear Nrf2 expression. (b-c) AMPK, p-AMPK, and nuclear Nrf2 quantification analysis. *N* = 3, ^*∗*^*P* < 0.05 vs. control. #*P* < 0.05 vs. H/R.

**Figure 5:** Effect of AMPK inhibition on PF-mediated Nrf2 signaling pathway activation in H/R induced H9c2 cells. H9c2 cells were exposed to H/R damage after being treated with PF in the presence of Compound C (10 M). (a) Western blot analysis of AMPK and Nrf2 nuclear protein expression. (b-c) P-AMPK and Nrf2 quantification analysis. (d) Cell viability in H9c2 cells. (e) ROS generation in H9c2 cells. (f) Caspase-3 activity in H9c2 cells, ^*∗*^*P* < 0.05 vs. control. #*P* < 0.05 vs. H/R, $*P* < 0.05 vs. H/R + PF group.

## Data Availability

The data used to support the findings of this study are available from the corresponding author upon request.
